The article "Application Effect of Laparoscopic Myomectomy and Comprehensive Rehabilitation Nursing on Patients with Uterine Fibroids" was published in 2022. Journal: Comput Math Methods Med.

# Application Effect of Laparoscopic Myomectomy and Comprehensive Rehabilitation Nursing on Patients with Uterine Fibroids

**DOI:** 10.1155/2022/4018803

**Published:** 2022-09-22

**Authors:** Zhihong Liu, Zhiwen Gao, Fangwei Li, Lifen Xu, Xinghua Liu

**Affiliations:** ^1^Department of Obstetrics and Gynecology, Zunhua People's Hospital, Hebei, China; ^2^Department of Obstetrics and Gynecology, Zhengding Maternal and Child Health Hospital, Shijiazhuang, Hebei, China; ^3^Department of Obstetrics and Gynecology, Anxin County Hospital, Xiguan Street, Anxin County, Baoding, Hebei, China

## Abstract

**Background:**

Uterine fibroids are most common in women aged 30-50 and are the most common benign gynecological tumors. Relevant data suggest that about 25% of patients with uterine fibroids are at childbearing age. Uterine fibroids not only cause the discomfort symptoms, and affect the pregnancy, but also have certain malignant transformation risk, thus needed to be treated positively and promptly.

**Aim:**

This study is aimed at exploring the effect of laparoscopic myomectomy and comprehensive rehabilitation nursing on patients with uterine fibroids.

**Methods:**

The clinical data of 110 cases of uterine fibroids admitted to our hospital from August 2019 to December 2021 were analyzed retrospectively, and they were divided into two groups according to postoperative rehabilitation strategies. Both groups were treated with laparoscopic myomectomy. The A group was treated with routine rehabilitation strategy, while the B group was treated with comprehensive rehabilitation nursing strategy. The differences in operation-related indicators, stress factors, inflammatory factors, nutritional indicators, knowledge mastery, occurrence of adverse symptoms and pain scores, negative emotion scores, nursing satisfaction, and simplified comfort status scale (GCQ) scores between the two groups under nursing strategies were compared.

**Results:**

The postoperative exhaust time (13.14 ± 2.03) h, bed time (9.86 ± 1.94) h, postoperative hospital stay (4.37 ± 1.31) d, and total hospital stay (6.78 ± 1.69) d in the B group were shorter than those in the A group, and the hospitalization expenses (0.74 ± 0.25) million were less than those in the A group (*P* < 0.05). Before operation, stress factors, inflammatory factors, and nutritional indexes were compared between the two groups (*P* > 0.05). On the 3rd day after operation, tumor necrosis factor-*α* (TNF-*α*), cortisol (Cor), norepinephrine (NE), and interleukin-1*β* (IL-1*β*) in the two groups showed a significantly upward trend compared with those before operation, and albumin and transferrin were significantly fell compared with those before operation. However, the values of stress factor and inflammatory factor in the B group were significantly lower than those in the A group, and the values after the decrease of nutritional index were significantly higher than those in the A group (*P* < 0.05). The pain scores at 24 h, 48 h, and 72 h after operation in the B group were significantly lower than those in the A group (*P* < 0.05). Negative emotions, nursing satisfaction, and GCQ scores were compared between the two groups before intervention (*P* > 0.05). After the intervention, the scores of Hamilton Depression Scale (HAMD) and Hamilton Anxiety Scale (HAMA) in the two groups were significantly lower than those before the intervention, and the scores of nursing satisfaction and GCQ were higher than those before the intervention. The values of negative emotions in the B group after the decline were significantly lower than those in the A group, while the values of nursing satisfaction and GCQ after the increase were higher than those in the A group (*P* < 0.05). The excellent and good rate of knowledge acquisition in the B group was 94.55% (52/55), which was significantly higher than 78.18% (43/55) in the A group (*P* < 0.05). The incidence of adverse symptoms in the B group was 9.09% (5/55), which was lower than 21.82% (12/55) in the A group, while the difference was not statistically significant (*P* > 0.05).

The article "Application Effect of Laparoscopic Myomectomy and Comprehensive Rehabilitation Nursing on Patients with Uterine Fibroids" was published in 2022. Journal: Comput Math Methods Med.

**Conclusion:**

Laparoscopic myomectomy combined with comprehensive rehabilitation nursing can reduce the postoperative stress state of patients with uterine fibroids, improve patient satisfaction, reduce adverse emotions, and promote rehabilitation.

## 1. Introduction

Uterine fibroids are common benign tumors in the female reproductive system, which can give rise to abnormal uterine bleeding, abdominal mass, abdominal pain, bulge, leucorrhea, infertility, abortion, and other symptoms and signs [1]. The etiology and pathogenesis of uterine fibroids have not been fully clarified so far. Mutations in myometrium cells, disorder of sex hormones, and abnormal local growth factors are thought to be related to the occurrence of this disease [2]. At present, surgical treatment is generally used in clinical practice to cause myomectomy, and laparoscopic myomectomy is one of the common surgical methods [3]. However, due to the impact of uterine fibroids disease itself and surgical trauma, the patient' s body is in a state of stress and cause negative emotions [4].

Nursing is an important supplement to clinical medical work. The implementation of high-quality nursing intervention after laparoscopic myomectomy helps to reduce the negative emotions of patients and actively cooperate with follow-up treatment [5]. Comprehensive rehabilitation nursing is a kind of comprehensive nursing intervention mode, starting from basic nursing, psychological counseling, health education, and other aspects to help patients recover better and return to normal work and life soon [6, 7]. This study explored the application effect of laparoscopic myomectomy and comprehensive rehabilitation nursing on patients with uterine fibroids, which is reported as follows.

The article "Application Effect of Laparoscopic Myomectomy and Comprehensive Rehabilitation Nursing on Patients with Uterine Fibroids" was published in 2022. Journal: Comput Math Methods Med.

Core tips were as follows: laparoscopic myomectomy is commonly used in the clinical treatment of uterine fibroids, and most patients can benefit from it. However, there are still a considerable number of patients with severe postoperative negative emotions, which is harmful to their recovery. In this study, patients with laparoscopic myomectomy were taken as the subjects to explore the impact of comprehensive rehabilitation nursing on their prognosis. It was found that laparoscopic myomectomy combined with comprehensive rehabilitation nursing can reduce the body stress state of patients with uterine fibroids after operation, improve patient satisfaction, reduce bad emotions, and promote rehabilitation.

## 2. Data and Methods

### 2.1. General Information

The data of 110 cases of uterine fibroids admitted to the hospital from August 2019 to December 2021 were analyzed retrospectively. The age was 22–43 years old, with an average of (35.45 ± 3.88) years old. According to the postoperative rehabilitation strategy, they were divided into two groups. The control group (group A) accepted the conventional rehabilitation strategy, and the observation group (group B) accepted comprehensive rehabilitation nursing strategy. The data between the two groups were balanced (*P* > 0.05), see Table 1

The inclusion criteria were as follows: (1) clinical diagnosis of uterine fibroids confirmed by enhanced MRI and ultrasonography [8]; (2) accompanied by menstrual abnormalities, abdominal pain, frequent urination, anemia, and other clinical symptoms; (3) The International Union of Obstetrics and Gynecology is classified as 0-VI [8]; (4) patients have indications for surgery, laparoscopic myomectomy was performed under general anesthesia, and the pathological results were leiomyoma of uterus; (5) complete clinical data and follow-up data; and (6) ages 18~45 years old.

The exclusion criteria were as follows: (1) there were coagulation abnormalities, such as platelet 25 s and prothrombin activity < 40%; (2) perimenopausal signs; (3) malignant lesions such as cervical cancer and endometrial cancer; (4) there is language communication disorder or cognitive dysfunction, unable to carry out effective communication or curative effect evaluation; (5) functional insufficiency of the liver and kidney; (6) self-injury, suicidal tendencies, or behavior; conversion to laparotomy; and (7) past history of abdominal and pelvic surgery.

The article "Application Effect of Laparoscopic Myomectomy and Comprehensive Rehabilitation Nursing on Patients with Uterine Fibroids" was published in 2022. Journal: Comput Math Methods Med.

### 2.2. Method

Patients in the two groups were treated with laparoscopic myomectomy and general anesthesia with tracheal intubation, and the patients were in supine position. A 10 mm incision was made at the upper edge of the umbilical wheel as the observation hole to establish pneumoperitoneum, and the pressure was maintained at about 12 mmHg. Laparoscopic exploration of abdominal cavity observes the number, size, and location of fibroids. Make a transverse incision on the toe joint and place the surgical instruments. The subserous myoma was ligated at the pedicle of the myoma, the myoma was removed at 5 mm above the ligation site, and the wound was electrocoagulation to stop bleeding. Intramyometrial myoma was injected with oxytocin at the most prominent part of the tumor. The myometrium of the uterus was cut to the fibroid capsule layer, and the fibroid nodules were stripped. The tumor cavity was closed by absorbable intestinal line. After determining no active bleeding, the abdominal cavity was washed, and sodium hyaluronate was injected to prevent intrauterine adhesions.

The A group accepted the conventional rehabilitation strategy. The patients were instructed to complete the preoperative examination before operation, and the operation precautions were informed by the visit. The patients were instructed to have reasonable diet, activities, and follow-up treatment according to the doctor's advice after operation.

The B group accepted comprehensive rehabilitation nursing strategy: preoperative psychological counseling, inform patients of the purpose of preoperative preparation, guide patients to pay attention to rest, and strengthen nutrition; according to the patient' s educational level, use comprehensive language to introduce the advantages of laparoscopic myomectomy and perioperative cooperation points. Guide patients to bed position and deep breathing training. Patients were asked to stay in bed absolutely for at least 24 h, drink more water, and eat light and digestible food on the day after operation. If the symptoms of limb numbness, pain, nausea, vomiting, fever occured, the nurse would tell them that these were normal reactions after operation to let them relaxed, and give symptomatic treatment. From the second day after operation, the patients were instructed to get out of bed properly, eat general food, and strengthen nutrition. Guide patients to take a comfortable position and relax the abdominal muscles, through chat, watch TV, and other methods to distract attention, to relieve pain. Severe pain can be given analgesics according to the doctor' s advice. Guide patients to rest after discharge, strengthen nutrition, maintain personal hygiene, avoid severe activity, and review on time. If the patients appeared abdominal pain, bleeding, etc.,the nurse would give timely treatment.

The article "Application Effect of Laparoscopic Myomectomy and Comprehensive Rehabilitation Nursing on Patients with Uterine Fibroids" was published in 2022. Journal: Comput Math Methods Med.

### 2.3. Observation Indicators and Detection Methods

The differences in operation-related indicators, stress factors, inflammatory factors, nutritional indicators, knowledge mastery, occurrence of adverse symptoms and pain scores, negative emotion scores, nursing satisfaction, and simplified comfort status scale (GCQ) scores between the two groups under nursing strategies were compared.

5 mL fasting peripheral venous blood samples were collected before operation and 3 days after operation and were placed in vacuum to collect blood vessels. The blood was centrifuged within 1 hour, and the rotation speed was 3000 r/min. The centrifugal time was 10 min. Tumor necrosis factor-*α* (TNF-*α*), serum cortisol (Cor), norepinephrine (NE), and interleukin-1*β* (IL-1*β*) were detected by enzyme-linked immunosorbent assay. Albumin was detected by bromocresol green method; transferrin was detected by immunoturbidimetry. The kit is produced by Shanghai Enzyme Linked Biological Technology Co., Ltd., and the detection instrument is Merry RT-96A.

### 2.4. Score Standard

Degree of pain was as follows: according to the visual analogue scale (VAS) score [9], the score is 0-10 points, and the score range indicates no heavy pain.

Negative emotions were as follows: according to the evaluation of Hamilton Depression Scale (HAMD) and Hamilton Anxiety Scale (HAMA) [10], 17 items were used in the HAMD score in this study, with the score higher than 24 divided into severe depression and the score higher than 17 divided into moderate depression: more than 7 points for mild depression and the score below 7 points without depression. HAMA score more than 29 points of severe anxiety, more than 21 points for positive anxiety, and more than 14 points have anxiety, and more than 7 points may exist anxiety.

Nursing satisfaction was as follows: in the hospital self-made scale evaluation, covering the environment, medical staff business level, attitude, etc., score range is 0-100 points, and score range indicates the low-high nursing satisfaction.

GCQ score [11] was as follows: evaluation of comfort, including physiology, social culture, psychological spirit, and environment, covers 28 items, with a single score of 1–4 and a total score of 28–112. The score range indicates the low–high comfort.

The level of mastery of relevant knowledge was as follows: hospital self-made scale covers the pathophysiology of the disease, postoperative care, precautions, diet, etc. The score range is 0–100 points, of which over 90 points are excellent, over 80 points are good, over 60 points are general, and less than 60 points are poor.

The article "Application Effect of Laparoscopic Myomectomy and Comprehensive Rehabilitation Nursing on Patients with Uterine Fibroids" was published in 2022. Journal: Comput Math Methods Med.

### 2.5. Statistical Method

The data were processed by SPSS26.0. The normality and homogeneity of variance of measurement data were tested by *K*-*S* test and Levene test, respectively. The measurement data conforming to the standard were described by (^−^*χ* ± *s*). The *t*-test was used for comparison. The enumeration data were compared by *χ*^2^ test. The *χ*^2^ test of four-grid table or row×list was used.

## 3. Results

### 3.1. Differences in General Data between the Two Groups of Patients

In terms of general information such as age, BMI, course of disease, pregnancy, maximum myoma diameter, disease type, tumor location, marital status, and educational level, no statistical significance was found between the two groups after statistical test (*P* > 0.05), see Table 1.

### 3.2. Differences in Surgical-Related Indicators between the Two Groups

The postoperative exhaust time (13.14 ± 2.03) h, ambulation time (9.86 ± 1.94) h, postoperative hospitalization time (4.37 ± 1.31) d, and total hospitalization time (6.78 ± 1.69) d in the B group were shorter than those in the A group, and the hospitalization cost (0.74 ± 0.25) ten thousand was less than that in the A group (*P* < 0.05), see Table 2.

### 3.3. Differences in Stress Factors and Inflammatory Factors between the Two Groups

Before operation, the stress factors and inflammatory factors were not statistically different between the two groups (*P* > 0.05). On the 3rd day after operation, the levels of Cor, NE, TNF-*α*, and IL-1*β* in the two groups were significantly higher than those before operation, while the values of the above factors in the B group were significantly lower than those in the A group (*P* < 0.05), see Table 3.

### 3.4. Differences in Nutritional Indicators between the Two Groups

Before operation, the nutritional indexes were not statistically different between the two groups (*P* > 0.05). Three days after operation, albumin and transferrin in both groups were significantly decreased compared with those before operation, while the nutritional indexes in the B group were higher than those in the A group (*P* < 0.05), see Table 4.

### 3.5. Difference in Postoperative Pain between the Two Groups

The pain scores at 24 h, 48 h, and 72 h after operation in the B group were significantly lower than those in the A group (*P* < 0.05), see Table 5.

### 3.6. Differences of Negative Emotion, Nursing Satisfaction, and GCQ Score between the Two Groups

Before intervention, the negative emotion, nursing satisfaction, and GCQ score were not statistically different between the two groups (*P* > 0.05). After the intervention, the HAMD score and HAMA score of the two groups were significantly lower than those before the intervention, and the nursing satisfaction score and GCQ score were higher than those before the intervention. The negative emotion of the B group was significantly lower than that of the A group, while the nursing satisfaction score and GCQ score were higher than those of the A group (*P* < 0.05), see Table 6.

The article "Application Effect of Laparoscopic Myomectomy and Comprehensive Rehabilitation Nursing on Patients with Uterine Fibroids" was published in 2022. Journal: Comput Math Methods Med.

### 3.7. Differences in Mastery of Relevant Knowledge between the Two Groups

The excellent and good rate of knowledge acquisition in the B group was 94.55% (52/55), which was significantly higher than 78.18% (43/55) in the A group (*P* < 0.05), see Table 7.

### 3.8. Difference in Occurrence of Adverse Symptoms between the Two Groups

The incidence of adverse symptoms in the B group was 9.09% (5/55), which was lower than 21.82% (12/55) in the A group, while the difference was not statistically significant (*P* > 0.05), see Table 8.

## 4. Discussion

In recent years, minimally invasive techniques have been widely used in the treatment of gynecological diseases. Traditional open myomectomy has gradually been replaced by laparoscopic surgery [12]. Laparoscopic surgery has the advantages of small wound, light pain and rapid postoperative recovery, but there are also complications such as pelvic adhesions and cervical stump bleeding. Due to little knowledge of laparoscopic surgery and uterine fibroids, patients have obvious perioperative negative emotions and poor psychological resilience [13, 14]. Routine nursing often only pays attention to the treatment of diseases, but not to the negative emotions and rehabilitation quality of patients [15].

Comprehensive rehabilitation nursing is a comprehensive nursing intervention model, involving medication, diet, exercise, psychology and other aspects of patients [16]. This study found that the postoperative exhaust time, ambulation time, postoperative hospitalization time and total hospitalization time of the comprehensive rehabilitation nursing intervention group were shorter than those of the routine nursing intervention group, and the hospitalization expenses were less than those of the routine nursing intervention group. The incidence of adverse symptoms was apparently lower than that of routine nursing intervention. This result suggested that laparoscopic myomectomy combined with comprehensive rehabilitation nursing could accelerate the postoperative rehabilitation process of patients and reduce adverse symptoms medical costs. This is due to the comprehensive rehabilitation nursing mode could make patients understand the operation process and rise perioperative cooperation points by preoperative psychological counseling and health education, thus better cooperating with the operation of medical staff. By guiding patients with reasonable diet, comprehensive rehabilitation nursing mode could promote wound healing and gastrointestinal function recovery, so as to accelerate the recovery process [17, 18].

The article "Application Effect of Laparoscopic Myomectomy and Comprehensive Rehabilitation Nursing on Patients with Uterine Fibroids" was published in 2022. Journal: Comput Math Methods Med.

Postoperative pain is an adverse factor affecting the compliance of patients with rehabilitation treatment, and can aggravate negative emotions and sleep disorders. Negative emotions and sleep disorders can increase the sensitivity of pain and cause pain. Severe pain can cause irritability and raise the risk of nurse-patient disputes [19, 20]. In this study, the pain score of patients 24 h, 48 h, 72 h after the operation were analyzed, and it was found that the comprehensive rehabilitation nursing intervention VAS score at each time point were considerably lower than the conventional nursing intervention; after intervention, HAMD and HAMA scores were lower than those of routine nursing intervention, and nursing satisfaction score, GCQ score and excellent rate of related knowledge mastery were higher than those of routine nursing intervention. The above results suggested laparoscopic myomectomy combined with comprehensive rehabilitation nursing could increase the comfort and satisfaction of patients, and enhance the mastery of relevant knowledge and reduce adverse emotions. This is due to the comprehensive rehabilitation nursing mode reduce the negative emotions of patients through psychological counseling, so that they can deal with the disease with a more optimistic and positive attitude. Health education deepens patients' understanding of disease-related knowledge and enhances their self-care ability. By guiding the patient to take a comfortable position, relax the abdominal muscle, chat, watch TV and other methods to distract attention, in order to alleviate pain. Severe pain can be given analgesics according to the doctor' s advice, so that patients with postoperative pain greatly reduced [21–23].

Surgical trauma can lead to stress response and inflammatory response in the body. Cor and NE are common clinical stress indicators, and the change of serum level can reflect the degree of stress response in the body [24–26]. TNF-*α* and IL-1*β* are classical inflammatory factors, which can influence and promote each other, and cause the expansion of inflammatory response [27–29]. Good nutritional status is an important prerequisite for promoting wound healing and rehabilitation of patients. Albumin and transferrin are commonly used clinical nutritional indicators. Patients with uterine fibroids are often in malnutrition due to abnormal uterine bleeding and intraoperative bleeding [30–32]. In this study, through the detection of the above indicators, it was found that the Cor, NE, TNF-*α* and IL-1*β* of the comprehensive rehabilitation nursing intervention group were higher than those of the routine nursing intervention group at 3d after operation, and the albumin and transferrin were evidently higher than those of the routine nursing intervention group. These results suggested that laparoscopic myomectomy combined with comprehensive rehabilitation nursing could relieve stress state and inflammatory response state of patients with uterine fibroids after operation, and improve the nutritional state of the body, which was an important mechanism for promoting postoperative rehabilitation of patients. Under the comprehensive rehabilitation nursing mode, psychological counseling enables patients to have a psychological preparation for the operation process and possible symptoms such as limb numbness, pain, nausea, vomiting and fever after operation, so as to reduce the stress response. Early postoperative guidance of patients with reasonable activity, take comfortable position to reduce the stress response caused by pain. Guiding patients to take a reasonable rest, avoiding intensive activities and increasing nutritional intake can improve the nutritional status of the body [33–35].

The article "Application Effect of Laparoscopic Myomectomy and Comprehensive Rehabilitation Nursing on Patients with Uterine Fibroids" was published in 2022. Journal: Comput Math Methods Med.

In summary, laparoscopic myomectomy combined with comprehensive rehabilitation nursing can reduce the body stress state of patients with uterine fibroids after operation, improve patient satisfaction, reduce adverse emotions, and promote rehabilitation.

## Figures and Tables

**Table 1:** Differences in general information between the two groups of patients.

Normal information	A group (*n* = 55)	B group (*n* = 55)	*χ* ^2^ or *t*	*P*
Age ($\left(\bar{\chi }\pm s\right)$, age)	35.27 ± 4.55	35.52 ± 4.18	0.300	0.765
BMI ($\left(\bar{\chi }\pm s\right)$, kg/m^2^)	22.56 ± 2.47	22.49 ± 2.51	0.147	0.883
Course of disease ($\left(\bar{\chi }\pm s\right)$, moon)	11.25 ± 3.75	11.09 ± 3.82	0.222	0.825
Pregnancy ($\left(\bar{\chi }\pm s\right)$, number)	1.78 ± 0.59	1.81 ± 0.63	0.258	0.797
Maximum fibroid diameter ($\left(\bar{\chi }\pm s\right)$, mm)	5.46 ± 0.31	5.51 ± 0.36	0.537	0.593
Disease type (*n* (%))			0.629	0.428
Single shot	33 (60.00)	37 (67.27)		
Multiple	22 (40.00)	18 (32.73)		
Tumor location (*n* (%))			0.037	0.848
Uterine submucosal fibroids	30 (54.55)	29 (52.73)		
Cervical fibroids	25 (45.45)	26 (47.27)		
Marital status (*n* (%))			0.367	0.545
Married	35 (63.64)	38 (69.09)		
Unmarried	20 (36.36)	17 (30.91)		
Educational level (*n* (%))			0.607	0.738
Elementary school and below	14 (25.45)	12 (21.82)		
Junior high school to high school	21 (38.18)	25 (45.45)		
College and above	20 (36.36)	18 (32.73)		

The article "Application Effect of Laparoscopic Myomectomy and Comprehensive Rehabilitation Nursing on Patients with Uterine Fibroids" was published in 2022. Journal: Comput Math Methods Med.

**Table 2:** Differences in surgery-related indicators between the two groups $\left(\bar{\chi }\pm s\right)$.

Group	*n*	Postoperative exhaust time (h)	Time to get out of bed (h)	Hospital stay (d)		Hospital costs (ten thousand)
				Postoperative hospital stay	Total hospital stay	
A group	55	15.89 ± 2.11	12.88 ± 2.19	5.24 ± 1.56	8.46 ± 1.83	0.86 ± 0.29
B group	55	13.14 ± 2.03	9.86 ± 1.94	4.37 ± 1.31	6.78 ± 1.69	0.74 ± 0.25
*t*		6.965	7.655	3.167	5.002	2.324
*P*		0.000	0.000	0.002	0.000	0.022

**Table 3:** Differences in stress factors and inflammatory factors between the two groups (*χ* ± *s*).

Group	*n*	Cor (ng/mL)		NE (ng/mL)		TNF-*α* (ng/mL)		IL-1*β* (*μ*g/L)	
		Preoperative	3 d after surgery	Preoperative	3 d after surgery	Preoperative	3 d after surgery	Preoperative	3 d after surgery
A group	55	131.54 ± 38.85	182.56 ± 34.17	301.52 ± 37.85	369.89 ± 41.75^∗^	13.52 ± 3.17	28.96 ± 4.52^∗^	7.89 ± 2.17	13.89 ± 2.57
B group	55	128.74 ± 42.16	153.69 ± 29.99	289.76 ± 41.07	331.25 ± 34.51^∗^	13.48 ± 3.69	22.54 ± 3.26^∗^	8.02 ± 2.24	11.75 ± 2.26
*t*		0.362	4.709	1.562	5.290	0.061	8.543	0.309	4.637
*P*		0.718	0.000	0.121	0.000	0.951	0.000	0.758	0.000

^∗^ represents the comparison with preoperative, *P* < 0.05.

**Table 4:** Differences in nutritional indicators between the two groups (^−^*χ* ± s).

Group	*n*	Albumin (mg/L)		Transferrin (g/L)	
		Preoperative	3 d after surgery	Preoperative	3 d after surgery
A group	55	369.98 ± 41.17	228.59 ± 36.69^∗^	2.25 ± 0.29	1.46 ± 0.25^∗^
B group	55	372.45 ± 36.52	254.56 ± 38.52^∗^	2.23 ± 0.31	1.68 ± 0.29^∗^
*t*		0.333	3.620	0.349	4.261
*P*		0.740	0.000	0.727	0.000

^∗^ represents the comparison with preoperative, *P* < 0.05.

**Table 5:** Differences in postoperative pain levels between the two groups (^−^*χ* ± *s*).

Group	*n*	VAS score (point)			
		6 hours after surgery	24 hours after surgery	48 hours after surgery	72 hours after surgery
A group	55	2.89 ± 0.47	3.48 ± 0.45	3.96 ± 0.41	2.58 ± 0.56
B group	55	2.91 ± 0.44	3.06 ± 0.37	3.38 ± 0.38	2.17 ± 0.39
*t*		0.230	5.347	7.695	4.456
*P*		0.818	0.000	0.000	0.000

**Table 6:** Differences in negative emotions, nursing satisfaction, and GCQ scores between the two groups ((^−^*χ* ± *s*), point).

Group	*n*	HAMD score		HAMA score		Nursing satisfaction score		GCQ score	
		Before intervention	After intervention	Before intervention	After intervention	Before intervention	After intervention	Before intervention	After intervention
A group	55	22.85 ± 4.15	16.96 ± 3.28^∗^	22.15 ± 3.96	17.23 ± 3.41^∗^	58.89 ± 7.47	74.88 ± 6.36^∗^	54.85 ± 8.14	71.54 ± 7.56^∗^
B group	55	23.03 ± 3.92	13.89 ± 3.11^∗^	22.04 ± 4.05	14.58 ± 2.86^∗^	60.75 ± 8.26	87.49 ± 6.17^∗^	53.74 ± 7.67	86.32 ± 8.07^∗^
*t*		0.234	5.037	0.144	4.416	1.239	10.554	0.736	9.912
*P*		0.816	0.000	0.886	0.000	0.218	0.000	0.463	0.000

^∗^ represents the comparison with preoperative, *P* < 0.05.

The article "Application Effect of Laparoscopic Myomectomy and Comprehensive Rehabilitation Nursing on Patients with Uterine Fibroids" was published in 2022. Journal: Comput Math Methods Med.

**Table 7:** Differences in the level of related knowledge mastery between the two groups.

Group	*n*	Excellent	Good	Generally	Difference	Excellent and good rate
A group	55	30 (54.55)	13 (23.64)	7 (12.73)	5 (9.09)	43 (78.18)
B group	55	46 (83.64)	6 (10.91)	2 (3.64)	1 (1.82)	52 (94.55)
*χ* ^2^						6.253
*P*						0.012

**Table 8:** Differences in the occurrence of adverse symptoms between the two groups.

Group	*n*	Urinary retention	Upset stomach	Urinary tract infection	Local edema	Wound infection	Total
A group	55	4 (7.27)	2 (3.64)	3 (5.45)	2 (3.64)	1 (1.82)	12 (21.82)
B group	55	1 (1.82)	1 (1.82)	2 (3.64)	1 (1.82)	0 (0.00)	5 (9.09)
*χ* ^2^							3.409
*P*							0.065

## Data Availability

The datasets used and analyzed during the current study are available from the corresponding author upon reasonable request.
